RETRACTED

# The abnormal expression of chromosomal region maintenance 1 (CRM1)-survivin axis in ovarian cancer and its related mechanisms regulating proliferation and apoptosis of ovarian cancer cells

**DOI:** 10.1080/21655979.2021.2012416

**Published:** 2022-01-03

**Authors:** Jing Zhang, Xinyan Xu, Yongfeng Chen, Xiaoju Guan, Hong Zhu, Yuhong Qi

**Affiliations:** a Department of Gynecology, Urumqi Maternal and Child Health Hospital of Xinjiang Uygur, Urumqi, Xinjiang Uygur Autonomous Region, China; b Pathology Department, Urumqi Maternal and Child Health Hospital of Xinjiang Uygur, Urumqi, Xinjiang Uygur Autonomous Region, China

**Keywords:** Ovarian cancer, CRM1, survivin, proliferation, apoptosis

## Abstract

Ovarian cancer (OC) is the main type of cancer that affects the female reproductive system and has a high morbidity and mortality rate. This study aimed to explore the regulatory effect of the chromosomal region maintenance 1 (CRM1)-survivin axis on the progression of OC. Ovarian cancer cells were transfected with pcDNA3.1-survivin and short hairpin RNA (sh)-CRM1. Cell proliferation was analyzed by cell counting kit-8 (CCK8), 5-ethynyl-2´-deoxyuridine (EdU) staining, and colony formation assays. Apoptosis was detected using flow cytometry. Quantitative real-time polymerase chain reaction (qRT-PCR) and Western blotting were performed to analyze the expression of RNA and protein, respectively. qRT-PCR and prognostic correlation analyses revealed that CRM1 is highly expressed in OC cells and related to survival. The results of qRT-PCR, CCK8, colony formation test, EdU staining, flow cytometry, and Western blotting showed that CRM1 silencing inhibited the proliferation and colony formation of OVCAR 3 and SKOV3 cells and promoted cell apoptosis by promoting Caspase-3 activation. Survivin was positively regulated by CRM1 and promoted the development of OC. The results of the rescue experiment showed that overexpression of survivin reversed the inhibitory effect of CRM1 knockdown on the proliferation of ovarian cancer cells and its inhibitory effect on apoptosis. Our findings confirm the role of the CRM1-survivin signal transduction axis in OC by regulating the proliferation and apoptosis of OC cells, and may thus serve as a potential therapeutic target for OC.

## Introduction

Ovarian cancer (OC) remains the most common malignant tumor of the female reproductive system and is associated with high morbidity and mortality [1,2]. In recent years, the standardized treatment and full-process management of ovarian cancer have gradually been paid attention to, and the tremendous has been improved to some extent, but the clinical outcome is still poor. However, early symptoms, recurrence and metastasis lead to the failure of ovarian cancer therapy, and they are also the key factors leading to the death of patients [3]. But drug resistance and relapse are common. The 5-year survival rate of patients is less than 40% [4]. Therefore, it is particularly important to identify genes related to the biology of OC and explore the mechanism of OC invasion and metastasis to improve the diagnosis rate of OC and reduce the mortality of patients.

RETRACTED

Chromosomal region maintenance 1 (CRM1), also known as export protein 1 (XPO1), is a key regulator of cancer progression and mediates the export of proteins that are essential for growth regulation and tumor suppression [5]. The nuclear export protein, CRM1, plays an important role in tumor development and pathogenesis of immune diseases. Studies have shown that CRM1 is significantly upregulated in a variety of tumor types, especially liquid tumors, including lymphoma, leukemia, and myeloma [6]. Nuclear tumor suppressor factors mediated by CRM1 include p53, p21, nuclear phosphosmin (nucleophosmin, NPM), and nuclear factor kappa B inhibitor alpha (IκBα) [7]. *In vitro* and *in vivo* [8] knock down of CRM1 expression inhibited cell cycle progression and proliferation of OC cells. Survivin is the smallest member of the inhibitor of apoptosis (IAP) gene family and is widely expressed in colorectal cancer, pancreatic cancer, liver cancer, and other tumor tissues. In ovarian and kidney cancer, survivin increases the aggressiveness of tumors by promoting the epithelial-mesenchymal transition (EMT) of tumor cells [6], but the mechanism that controls its nuclear-cytoplasmic localization remains unclear. Consistent with a recent report describing the nuclear accumulation of survivin in gastric cancer cells [9], we detected survivin in the nucleus of lung cancer cells. Therefore, we hypothesized that CRM1 may affect the proliferation and apoptosis of OC cells by regulating survivin expression.

In our study, we aimed to find the role of CRM1 in OC and explore the molecular mechanism. CRM1 and survivin levels were highly expressed in OC cells. Through a series of functional and biochemical analyses, we found that CRM1 regulates the proliferation and apoptosis of OC cells by synergistically controlling the expression of survivin. This study provided a theoretical basis for CRM1-survivin axis as therapeutic target.

## Materials and methods

### Cell culture

Human OVCAR-3, Skov3, HOSE, CaOV-3 and ES-2 cell lines were obtained from the American Type Culture Collection (ATCC, Manassas, VA, USA). A2780 cells were acquired from European Collection of Cell Cultures (ECACC, Public Health England, UK). Cells were grown in Dulbecco’s Modified Eagle’s medium (DMEM, Gibco, Grand Island, NY, USA) (containing 10% fetal bovine serum, 1% penicillin and streptomycin, Hyclone, South Logan, UT, USA) and in an incubator at 37°C and 5% CO_2_.

RETRACTED

### Cell transfection

Survivin overexpression vector pcDNA3.1-survivin, short hairpin RNA (sh)-CRM1 and their negative controls were purchased from Sangon Biotech (Shanghai, China). Lipfectamine 2000 regent (Invitrogen, Carlsbad, CA, USA) was used to transfected pcDNA3.1-survivin into SKOV3 and OVCAR-3 following the protocols. Sh-CRM1 lentiviral plasmid and packaging plasmid were co-transfected into 293 T cells. After that, viral particles were acquired after ultracentrifugation. SKOV3 and OVCAR-3 cells were transfected with virus in complete medium containing polybrene. Forty-eight hours later, the culture medium was replaced by complete DMEM.

### Cell counting kit-8 (CCK8) analysis

CCK-8 analysis was performed similar with a previous study [10]. Cells were seeded on a 96-well plate and cultured in a 96-well microplate (Corning, Corning, NY, USA) at a concentration of 5 × 10^3^ cells /well. Then, the cells are transfected. When time is up, 10 μL CCK-8 reagent (Sigma, St. Louis, MO, USA) was added to each well, and then incubate for 2 h. A microplate reader (Bio-Rad, Hercules, CA, USA) was used to analyze the absorbance at 450 nm.

### Colony formation assay

Colony formation was conducted according to a previous study [11]. The OVCAR-3 and SKOV3 cells were seeded in 6-well plates at a concentration of 1 × 10^3^ cells/well and maintained at 37°C and 5% CO_2_ for 2 wks. Finally, the cells were fixed in 4% paraformaldehyde and stained with 0.5% crystal violet (Sigma) in methanol for 0.5 h. The number of colonies (>50 cells) was counted using a microscope.

### 5-ethynyl-2´-deoxyuridine (EdU) staining assay

EdU staining assay was conducted according to a previous study [12]. After transfection, the cells were treated with 20 mmol/L of EdU working solution for 2 h. The cells were then fixed in 4% paraformaldehyde for 20 min at 25°C. The EdU-positive cells in the different groups were then analyzed.

### Flow cytometry assay

Cell apoptosis was evaluated in line with a previous study [13]. Cells (1 × 10^5^ cells/mL) were cultured in Dulbecco’s modified Eagle’s medium (DMEM) containing 10% fetal bovine serum (FBS) in a 6-well plate for 24 h. Then the cells were stained with the Annexin V-PE (KeyGEN, Nanjing, China) staining kit according to the manufacturer’s instructions. Finally, the apoptotic cells were analyzed using a Verse Flow Cytometry System (BD Biosciences, San Jose, CA, USA).

### Western blotting

Total protein was extracted using radioimmunoprecipitation assay buffer (Jiancheng, Nanjing, China), separated by sodium dodecyl sulfate polyacrylamide gel electrophoresis (SDS-PAGE) for immunoblot assays. Membranes were blocked with 5% nonfat milk and then incubated with primary antibodies (anti-CRM1: ab24189; 1:500, anti-bax: ab182733; 1:2000, anti-bcl-2: ab182858; 1:2000, anti-cleaved Caspase-3: ab2302, 1:500, anti-survivin: ab76424, 1:10,000, anti-GAPDH: ab9485, 1:2500, Abcam, Cambridge, CA, USA) at 4°C overnight. Subsequently, the blots were incubated with horseradish peroxidase (HRP)-labeled secondary antibody (ab205718; 1:20,000, Abcam) for 2 h at room temperature. The protein bands were visualized with an enhanced chemiluminescence reagent and quantitated using ImageQuant LAS 4000 (GE Healthcare, Pittsburgh, Pennsylvania, USA).

RETRACTED

### Quantitative real-time polymerase chain reaction (qRT-PCR)

The total RNA was extracted using TRIzol reagent (Invitrogen). RNA (500 ng) was used to synthesize a cDNA template, PrimeScript RT kit (Takara, Beijing, China). The realtime PCR reaction was performed with a SYBR Green Mix kit (Jiancheng) and in an ABI7500 FAST system. The relative expression was calculated using 2^−ΔΔCt^ method.

### Statistical analysis

Each experiment was repeated three times. The results are presented as the mean ± standard deviation (SD). SPSS software (version 19.0) was used to analyze the data. The statistical significance of the comparison between the two or three groups was analyzed using Student’s *t*-test or one-way analysis of variance. Statistical significance was set at p < 0.05.

## Results

Herein, we investigated the role of CRM1-survivin axis in OC. We found CRM1 and survivin levels were increased in OC. Survivin was positively regulated by CRM1. Functionally, interfering CRM1 inhibited the proliferation, colony formation and facilitated apoptosis of OC cells by regulating survivin. These findings showed that CRM1 and survivin may be new OC therapeutic targets.

CRM1 was highly expressed in OC cells and was related to poor prognosis

Analysis of gene expression revealed that CRM1 levels were higher in the OC tissues than in the normal tissues (Figure 1a). Using the P values and hazard ratios of the R-package (when the optimal expression signal is cut off), the survival curve was determined. A higher CRM1 level was significantly associated with a poor prognosis (Figure 1b). qRT-PCR analysis of non-cancerous human ovarian surface epithelial (HOSE) cells and OC cell lines (OVCAR 3, SKOV3, CaOV-3, A2780, and ES-2) revealed that CRM1 was highly expressed in OC cell lines and was the highest in OVCAR 3 and SKOV3 cells (Figure 1c). Western blotting further confirmed that among HOSE cells and OC cell lines (OVCAR 3, SKOV3, CaOV-3, A2780, and ES-2), CRM1 protein level was highest in OVCAR 3 and SKOV3 cells (Figure 1c). These results indicate that elevated CRM1 expression plays an important role in the pathophysiology of OC.

RETRACTED

**Figure 1.** Expression of CRM1 in OC and its prognostic correlation. A, qRT-PCR was performed to assess CRM1 level in the normal and the OC groups. B, Kaplan-Meier diagram showing the prognostic correlation between CRM1 expression and overall survival of patients with OC. C, qRT-PCR was used to measure the mRNA level of CRM1 in OC cell lines. D, Western blotting was used to assess the protein level of CRM1 in OC cell lines. **P < 0.01 compared to the normal or HOSE group. OC: ovarian cancer, qRT-PCR: quantitative real-time polymerase chain reaction, HOSE: human ovarian surface epithelial cells.

Lentiviral transfection-mediated knock down of CRM1 reduced the proliferation rate of OC cells

Next, we sought to determine the role of CRM1 in the proliferation of OC cells. The results of qRT-PCR showed that transduction of OVCAR3 and SKOV3 cells with sh-CRM1 lentivirus significantly reduced the mRNA and protein expression of CRM1 (Figure 2a and b). The results of MTT assay showed that sh-CRM1 significantly inhibited the viability of OVCAR3 and SKOV3 cells (Figure 2c). Furthermore, colony formation test showed that the colony formation rate of the sh-CRM1 group was much lower than that of OVCAR3 and SKOV3 cells (Figure 2d). EdU analysis showed that sh-CRM1 treatment significantly reduced the number of EdU-positive cells (Figure 2e). These results indicate that sh-CRM1 inhibits the proliferation and colony formation of OVCAR 3 and SKOV3 cells.

**Figure 2.** Effect of CRM1 on proliferation of OVCAR3 and SKOV3 cells. A, qRT-PCR was used to detect the expression of CRM1 in OC cells following lentiviral transduction of sh-CRM1 into cells. B, Western blot was applied to determine the protein expressione of of CRM1 in OC cells following lentiviral transduction of sh-CRM1 into cells. C, CCK-8 was used to analyze the viability of OC cells following lentiviral transduction of sh-CRM1. D, Cell colony formation test was used to analyze the colony formation rate of OC cells following lentiviral transduction of sh-CRM1. E, EdU staining was used to detect the proliferation rate of OC cells following lentiviral transduction of sh-CRM1. **P < 0.01 compared to the NC group. OC: ovarian cancer, sh: short harpin RNA, CCK-8: cell counting kit-8, EdU: 5-ethynyl-2´-deoxyuridine, NC; negative control.

### Lentiviral transfection of sh-CRM1 induced apoptosis of OC cells

To evaluate whether CRM1 influences cell apoptosis, flow cytometry was performed. Compared with untreated cells, there was a significant increase in the apoptotic rate of sh-CRM1 transfected cells (Figure 3a). To further explore the mechanism by which CRM1 induces cell apoptosis, the expression of Caspase-3 was detected by Western blotting. The results showed that compared to the control cells, sh-CRM1 transfected cells showed significantly higher levels of cleaved Caspase-3. In addition, the expression level of bcl-2 was significantly reduced, while that of Bax was increased in sh-CRM1 transfected OC cells (Figure 3b and c). These data indicate that CRM1 silencing promotes cell apoptosis.

RETRACTED

**Figure 3.** Effect of CRM1 on apoptosis of OVCAR3 and SKOV3 cells. A, Flow cytometry was performed to evaluate the apoptotic rate of OC cells following lentiviral transduction of sh-CRM1. B, C Western blotting was used to detect the protein expression of bax, bcl-2, and cleaved Caspase-3 in OC cells following lentiviral transduction of sh-CRM1. **P < 0.01 compared to the NC group. OC: ovarian cancer, sh: short harpin RNA, NC; negative control.

### Expression of survivin in OC cells

Increasing evidence suggests that survivin is overexpressed in human cancers [14] and is involved in chemoresistance and metastatic progression [15]. In addition, CRM1 has been reported to be involved in the regulation of surviving [16]. To verify the role of survivin and the interaction between CRM1 and survivin in OC progression, we analyzed the expression of survivin following CRM1 knockdown. The qRT-PCR results indicated that following knockdown of CRM1, the expression of survivin in SKOV3 and OVCAR3 cells was significantly reduced (Figure 4a). Western blotting further confirmed that following CRM1 knockdown, the level of survivin in SKOV3 and OVCAR3 cells was significantly decreased in the OC cells compared to the normal cells (Figure 4b). Active transport between the nucleus and the cytoplasm may constitute an important regulatory mechanism of survivin function. The results of Western blot experiments indicated that following CRM1 knockdown, the levels of nuclear survivin were markedly elevated in SKOV3 and OVCAR3 cells, whereas CRM1 expression in the cytoplasm was reduced (Figure 4c). Gene expression analysis also indicated that the expression of survivin was increased in the OC cells compared to that in normal cells (Figure 4d). There was a significant positive correlation between the expression levels of CRM1 and survivin in OC (r2 = 0.7749, p = 0.001) (Figure 4e). These results indicate that survivin expression was regulated by CRM1.

**Figure 4.** CRM1 promotes the expression of survivin in OC cells. A, qRT-PCR was used to detect the level of survivin in OC cells following CRM1 knockdown. B, Western blotting was used to detect survivin protein level in OC cells following CRM1 knockdown. C, Western blotting was used to detect the levels of nuclear and cytosolic survivin in OC cells following CRM1 knockdown. D, qRT-PCR was used to compare the expression of survivin in cancer and normal tissues. E, Correlation analysis between the expression level of CRM1 and survivin in tumor tissues. **P < 0.01 compared to the NC or normal group. OC: ovarian cancer, qRT-PCR: quantitative real-time polymerase chain reaction, sh: short harpin RNA, NC; negative control.

RETRACTED

Overexpression of survivin reversed the inhibitory effect of CRM1 knockdown on the proliferation of OC cells.

To study the effect of CRM1 and the downstream tumor suppressor survivin, we overexpressed survivin following CRM1 knockdown. qRT-PCR experiments showed that in OC cells, survivin overexpression rescued the effect of CRM1 silencing (Figure 5a). MTT assay showed that in OC cells, overexpression of survivin reversed the CRM1 knockdown-mediated inhibitory effect on the viability of OC cells (Figure 5b). The results of colony formation experiments showed that survivin rescued the effect of CRM1 silencing on the colony formation rate of OC cells (Figure 5c). In addition, results of EdU analysis showed that overexpression of survivin reversed the inhibitory effect of CRM1 knockdown on the proliferation rate of OC cells (Figure 5d). These results indicate that overexpression of survivin reverses the inhibitory effect of CRM1 knockdown on the proliferation of OC cells.

**Figure 5.** Effect of overexpression of survivin on proliferation of OC cells. A, qRT-PCR results showing the level of survivin in OC cells following overexpression of survivin in cells with CRM1 knockdown. B, CCK8 experiment was used to detect the viability of OC cells following overexpression of survivin in cells with CRM1 knockdown. C. Colony formation experiment was used to detect the colony formation rate of OC cells following overexpression of survivin in cells with CRM1 knockdown. D, EdU staining was used to detect the proliferation rate of OC cells following overexpression of survivin in cells with CRM1 knockdown. **P < 0.01. OC: ovarian cancer, qRT-PCR: quantitative real-time polymerase chain reaction, CCK-8: cell counting kit-8, EdU: 5-ethynyl-2´-deoxyuridine.

Overexpression of survivin reversed the inhibitory effect of CRM1 silencing on apoptosis of OC cells

Flow cytometric analysis showed that survivin rescued the function of CRM1 silencing on the apoptosis of OC cells (Figure 6a). Western blotting revealed that overexpression of survivin reversed the effect of CRM1 knockdown on Caspase-3 activation in OC cells. As expected, survivin overexpression inhibited the expression of Bax and cleaved Caspase3 whereas it promoted the expression of bcl-2 compared to the CRM1-silenced group (Figure 6b). These results indicate that overexpression of survivin reverses the inhibitory effect of CRM1 knockdown on the apoptosis of OC cells.

RETRACTED

**Figure 6.** Effect of overexpression of survivin on apoptosis of OC cells. A, Flow cytometric analysis of the apoptosis rate of OC cells following overexpression of survivin in cells with CRM1 knockdown. B, Western blotting was used to analyze the expression of Caspase-3, Bax and Bcl-2 proteins in OC cells following overexpression of survivin in cells with CRM1 knockdown. **P < 0.01. OC: ovarian cancer.

## Discussion

According to global cancer data, 295,000 new cases of OC were diagnosed worldwide and 185,000 women died of OC in 2018. Surgery combined with chemotherapy remains the main treatment for OC. Although biological drug treatments targeting specific genes brings new hope to patients with OC, there is currently no evidence that OC can be cured [17,18]. The occurrence and development of OC are closely related to abnormalities in gene expression and tumor-related signaling pathways. Therefore, researchers have attempted to explore the etiology of OC from these perspectives to find new targets for its treatment. Increasing number of studies have shown that better understanding of disease pathogenesis and identification of biomarkers are helpful in early detection and treatment of OC [19,20].

CRM1 has recently been shown to be an effective drug target in a variety of cancers. Experiments have shown that knockdown CRM1 inhibits cell cycle and proliferation. Inhibition of CRM1 restores the nuclear localization and function of tumor suppressors, leading to cancer cell apoptosis [21,22]. CRM1 regulates the expression of proteins, including most tumor suppressor proteins such as FoxOs, p53, p21, p27, APC, survivin, and inhibitor of κB-α (IκB-α) [23]. Thus, CRM1 is involved in various signaling pathways at the same time, which makes it a promising therapeutic target for OC.

In this study, we have demonstrated that the expression of CRM1 is increased in OC cells compared to normal cells, and that higher CRM1 level is significantly associated with poor prognosis, consistent with a previous study [24]. The data suggested that CRM1 is a prognostic biomarker in OC and indicated that CRM1 plays an important role in the pathophysiological development of OC. Among the OC cells analyzed in the study, OVCAR-3 and SKOV showed the highest expression of CRM1, and therefore the subsequent experiments were carried out in these two cell types. Apoptosis is closely associated with tumor development [25], and Bax and Bcl-2 are the main factors that control apoptosis [26]. The ratio of Bax/Bcl-2 activity level, not the level of a single protein, is the key determinant of apoptosis sensitivity [27]. The caspase family is a key regulator of this process. The study showed that following lentiviral transfection-mediated knockdown of CRM1, the reduced the proliferation rate and induced apoptosis of OC cells. The expression of cleaved caspase-3 and Bax increased, whereas the expression of Bcl-2 decreased, and the ratio of Bax/Bcl-2 *in vitro* was significantly increased. These results showed that the apoptosis of OC cells was regulated by caspase-dependent apoptosis and Bax/Bcl-2 levels. Taken together, silencing of CRM1 attenuated the development of OC, suggesting that CRM1 has tumor promoting function, which is consistent with a previous study [28].

RETRACTED

Survivin is a kind of anti-apoptosis protein, who is involved in the pathogenesis, progression and metastasis of tumors [29]. Except apoptosis, it is also regulated other cellular processes, such as cell proliferation and invasion. Survivin plays a crucial role in numerous types of malignancies as an oncogene, such as bladder cancer and colorectal cancer [30,31]. In gynecological tumors, survivin causes cervical cancer cells to be sensitive to radiation treatment [32]. Additionally, survivin acts as a prognostic biomarker in breast cancer [33]. However, the role of survivin in OC is not fully understand.

In the present study, we also found that the expression level of CRM1 in OC was significantly related to the level of survivin. To verify the influence of survivin in regulating OC cell biofunction, we analyzed the effect of CRM1 and survivin on cell proliferation and apoptosis. We overexpressed survivin in cells following CRM1 knockdown and found that overexpression of survivin reversed the inhibitory effect of CRM1 knockdown on the proliferation and apoptosis of OC cells. The data suggested that silencing of CRM1 alleviated the progression of OC via decreasing survivin expression.

## Conclusions

In summary, highly expressed CRM1 was found in OC and related to poor prognosis. Survivin was regulated by CRM1. CRM1 accelerated cell proliferation and suppressed apoptosis via survivin in OC cells. These findings provide a novel understanding of OC development as well as new therapeutic targets for OC.

## Highlights

1. CRM1 was highly expressed in OC tissues and cells.

2. A loss of CRM1 inhibited the proliferation, colony formation and induced apoptosis.

3. Survivin was highly expressed in OC tissues and positively related to CRM1.

4. Suppression of CRM1-survivin axis attenuated the progression of OC.
